The article "Hotel Review Classification Based on the Text Pretraining Heterogeneous Graph Neural Network Model" was published in 2022. Journal: Comput Intell Neurosci.

# Hotel Review Classification Based on the Text Pretraining Heterogeneous Graph Neural Network Model

**DOI:** 10.1155/2022/5259305

**Published:** 2022-03-08

**Authors:** Liyan Zhang, Jingfeng Guo, Rui Kang, Bo Zhao, Chunying Zhang, Jia Li

**Affiliations:** ^1^College of Information Science and Engineering, Yanshan University, Qinhuangdao, Hebei, China; ^2^School of Science, North China University of Science and Technology, Tangshan, Hebei, China

## Abstract

With the amount of online information continuously growing, it becomes more and more important for online stores to recommend corresponding products precisely based on users' preferences. Reviews for various products can be of great help for the recommendation task. However, most recommendation platforms only classify positive and negative reviews based on sentiment analysis, without considering the actual demands of users, and it will reduce the effectiveness on classification task. To count this issue, we propose a new model, which integrates heterogeneous neural network and text pretraining model into this task, and compare this model with others on a travel type classification task. The model combines a pretrained text model named Bidirectional Encoder Representation from Transformers (BERT) and heterogeneous graph attention network (HGAN). Firstly, we do a fine-tuning task on BERT by a dataset consisting of 1.4 million hotel reviews from the Ctrip website to obtain fine representations of trip-related words. Then, we proposed the similarity fussy-matching method to get the main topic of each review. Then, we construct a heterogeneous neural network and apply the attention mechanism to it to mine the preference of users for traveling. Finally, the classification task is done based on each user's preference. In Section 5 of this study, we do an experiment, which compares our model with five others. The results show that the accuracy of ours is 70%, which is higher than the other five models.

## 1. Introduction

Online reviews are becoming important references for customers to obtain information and make decisions. It is particularly important to organize and manage massive data efficiently [1]. Due to the fast development of the online service, people who are planning to travel have been used to reference the opinions of other travelers while making traveling decisions on choosing hotels and tourist spots. However, confronting a variety of recommended options, users will have to spend a large amount of time to get enough information to get over this problem. So, mining users' preferences from massive information and then recommending the most related reviews to users based on their needs are urgent need to reduce users' information-digestion time and then improve the user experience.

The article "Hotel Review Classification Based on the Text Pretraining Heterogeneous Graph Neural Network Model" was published in 2022. Journal: Comput Intell Neurosci.

Review classification can be divided into several different problems according to different goals, such as topic classification and sentiment classification [2]. Currently, researches about online review classification focus on text sentiment analysis [3], topic classification, and review usefulness analysis [4–7]. Most studies apply this technique to the field of hotel management [8–10], but rarely mine users' preferences according to contents of reviews and make review classification according to the actual demands of users. However, most text classification methods are proposed with respect to English datasets. Compared with English, Chinese text has different linguistic features, and word segmentation is more difficult. Moreover, there are so many polysemy and ambiguous meanings of one word, which undoubtedly increases the difficulty of text analysis. It is difficult for traditional algorithms to work well and train efficiently on a large dataset containing amounts of text reviews.

A heterogeneous information network (HIN), a complex network composed of nodes and links of different types, is proposed on the basis of homogeneous network, which is studied for a long time. The containing information in the network is a lot more abundant, and this type of network can be utilized in the fields of natural language processing (NLP) with surprising performance. However, due to the colloquialization of review texts, the information conveyed by the content could be very few. So, making use of the heterogeneous network to mine as many features as possible can greatly benefit the job of short text classification.

In this study, we solved the problem that is labeling massive reviews by getting well-learned word representations through pretrained model, which helps us to avoid the amounts of time on labeling reviews of a large-scale dataset [11, 12].

Moreover, we proposed a hybrid model, which is as shown in Figure 1, and combined pretrained word representations learned using BERT and a heterogeneous graph neural network named heterogeneous graph attention network (HGAN) model. We also build a hotel review corpus in Chinese using Web crawling for this task and then processed to use the fuzzy similarity matching to build edges of heterogeneous networks to dig up different kinds of travel (different user demands) of user preference characteristics and classify reviews according to the characters of preference.

As shown in Figure 1, the preferences of users on travel types can be mined according to the reviews of other customers, and the results of review classification can be served to users as reasons for choosing a satisfying hotel with the only-known travel types of users. The model in this study can be applied to hotel recommendation system to assist users to make a better decision. Meanwhile, it can also help hotel managers to improve the service quality of hotels.

The article "Hotel Review Classification Based on the Text Pretraining Heterogeneous Graph Neural Network Model" was published in 2022. Journal: Comput Intell Neurosci.

To sum up, the main work of this study is as follows:

1. A hotel review corpus is established. The heterogeneous information network was constructed with travel type, review text, and topic words as nodes, and the Bidirectional Encoder Representation from Transformers (BERT)-heterogeneous graph attention network (HGAN) model was constructed by combining BERT and heterogeneous information network methods.
2. The hotel review content is predefined into seven categories of topics: location, catering, service, room, price, sanitation, and facilities. The fuzzy matching principle is proposed to identify the review topics and build edges of heterogeneous networks. The graph convolutional network (GCN) is adopted to complete the feature mapping of different nodes, and combined with the attention mechanism, the attention of different review texts to topic words and the attention of users of different travel types to different topic words are calculated from two perspectives, so as to obtain the user preference characteristics. Then, Chinese hotel reviews are classified according to user preferences of different travel types.

## 2. Related Work

Text is the information carrier with the widest distribution and the largest amount of data on the network. Accurate text classification can provide strong support for resource retrieval and personalized recommendation services such as news and information. Therefore, the problem of text classification has been concerned widely by researchers. As early as the 1970s, Salton et al. [13] proposed vector space model (VSM), which was successfully applied to the famous SMART system. In the following 50 years, text classification has been mainly based on shallow learning model, for example, naive Bayes-based text classification method, K-nearest neighbor method, and support vector machine method [14–16]. Although these methods have improved accuracy, they all rely on complex feature processing engineering and do not take into account the semantic information of the text. In 2013, Google proposed the open-source word vector calculation tool Word2vec [17], which takes into account the semantic information of the text and can predict words according to the context. Subsequently, the classic model transformer was proposed [18], which used self-attention mechanism to optimize the sequence structure of RNN, so that it can be trained in parallel and have global information. Based on the transformer model idea, in 2018, the Google AI team proposed pretraining of deep bidirectional transformers for language (BERT) based on bidirectional transformer understanding [19]. It can better complete downstream tasks such as classification and annotation and set a new record in multiple tasks.

The article "Hotel Review Classification Based on the Text Pretraining Heterogeneous Graph Neural Network Model" was published in 2022. Journal: Comput Intell Neurosci.

The short text is characterized by sparse semantics, low content information, and limited labeling data. Therefore, many researchers try to expand the content of short text by different methods. The commonly used text extension methods include the introduction of external corpus information [20] and the feature extension based on the short texts [21]. Shao Shao and Liu [22] combined the two methods and proposed a short text classification method based on category feature extension. With the continuous development of deep learning technology, researchers have also applied heterogeneous networks to text classification tasks. The key problem of using heterogeneous networks to do short text analysis is to utilize the complex network structure to expand the text content and integrate richer semantic information. Wang et al. [23] proposed the heterogeneous graph neural network model heterogeneous graph attention network (HAN) based on hierarchical attention. By learning the importance between nodes and neighbors, this model makes embedded representation of nodes and finally completes the task of text classification. Liang et al. [24] established a method based on graph neural network to do text classification (TextGCN). This model can capture the relationship between documents and words as well as global word co-occurrence information, enriching the semantic information of discontinuities and long distances in texts [25]. Hu et al. [26] proposed a new two-level attention mechanism (including node level and type level) to integrate topic (entities) into short texts and capture rich relationships between texts and between texts and additional information, thus alleviating the problem of sparse features in short texts and thus solving the problem of short text classification [27].

Based on the above work, it is not difficult to find that pretraining model and graph neural network model are the research hot spots of text classification task, but in practical application, pretraining-based model often needs fine-tuning process to obtain better classification effect. At the same time, the graph neural network model is limited by the lack of annotated text, and it is difficult to show its own advantages in large-scale datasets, so this study tries to merge the two algorithms. The pretraining model is used to get better text representation, and the heterogeneous graph neural network is used to expand the semantic information of the short text. Then, the user preference characteristics are mined, and the potential relationship between user preference and review text is mined from the perspective of different user needs of different travel types, and the review text is classified and recommended to users of different travel types.

The article "Hotel Review Classification Based on the Text Pretraining Heterogeneous Graph Neural Network Model" was published in 2022. Journal: Comput Intell Neurosci.

## 3. The Establishment of the BERT-HGAN Model

In the field of NLP, pretraining of language models has long been proved to be the best choice to improve the performance of downstream models. At present, the pretraining methods proposed can be divided into two types as follows:

1. The main feature-based representation was embeddings from language models (ELMO), which used the task model to learn the combination parameters of the internal implicit state of the pretrained language model
2. The main representative of fine-tuning is OpenAI GPT, which uses task data to fine-tune the trained language model

However, there is a problem in all the pretraining above; that is, in the pretraining process, only considering the one-way order of the text cannot learn the information of the lexical context well. Bidirectional Encoder Representations from Transformers (BERT) improved the bidirectional encoder representation from corpus using the masked language model based on fine-tuning. In this study, BERT is used to pretrain the crawling hotel reviews, and it is perfectly combined with the graph neural network model to improve the classification effect. A fuzzy similarity matching method is proposed to identify the theme corresponding to the review, and a heterogeneous network is constructed. An attention mechanism is added to the graph neural network to mine the preference and attention of users of different travel types on the review theme, and then, the hotel review is classified according to the user preference, as shown in Figure 2.

### 3.1. Dataset Analysis

As this study mainly addresses the classification of hotel reviews, the model interpretation takes this problem as an example.

This article uses a Web crawler to obtain 1.4 million hotel user reviews from 5000 hotels on the Ctrip website. In these reviews, users travel in five types, including solo travel, family travel, friends travel, couples travel, and business travel.

Through the analysis of the dataset, it is concluded that different types of travel users have different needs for hotels. For example, single travel users who travel with friends have different demands for hotel facilities and room types, but may have the same needs as other single travelers. Family travel users and business travel users also have different demands. Therefore, in the face of review information, readers are more inclined to choose reviews with the same demands as their own as a reference. Therefore, the type of travel is an important factor in hotel recommendation, and the hotel reviews given by users of different travel types represent the user preferences of different demands.

The article "Hotel Review Classification Based on the Text Pretraining Heterogeneous Graph Neural Network Model" was published in 2022. Journal: Comput Intell Neurosci.

To dig the preference characteristics of users with different travel types from the reviews and the potential relationship between user demands and hotel reviews, in this study, we first perform Jieba word segmentation on these reviews and verify them. Words that do not contribute much to the review classification are added to the stop word database for stop word filtering [28]^.^ At last, we make word frequency statistics on these reviews according to the types of travel, and the visual results are shown in Figure 3.

As can be seen from Figure 3, most of the users focus on the hotel room, service, and breakfast. To explore the attention degree of different *t* travel types to different topics of hotel services, this study establishes a topic word index based on a fuzzy matching algorithm to identify the topics mentioned in the reviews.

### 3.2. Fuzzy Matching of Review-Related Topic Words

First, the hotel's service topics are booked into seven categories: location, catering, service, room, price, sanitation, and facilities. Then, all word vector representations are obtained according to the Bert model, and the similarity is solved with the word vector representations of the seven topics. Finally, the top 15 topic words that are most relevant to these seven topics are calculated. (It can be seen from Figure 4 that the classification effect is best when the number of subject words is 15, so top 15 subject words are selected here.) The extraction results are shown in Table 1: location, catering, service, room, price, cleanliness, and facilities.

Taking the topic of services as an example, the topic words related to the service theme are as follows: (politeness 0.7029, politeness 0.6435, attitude 0.6404, friendliness 0.59159, enthusiasm 0.5838, politeness 0.5479, service 0.5393, friendliness 0.5211, friendliness 0.50903, enthusiasm 0.5080, service in place 0.4971, responsive 0.4861, quality 0.4780, warm heart 0.4748, and hospitality 0.4682).

### 3.3. Establishment of the Heterogeneous Graph Neural Network

To dig the preference characteristics of users from the reviews, that is the potential relationship between users' demands and hotel reviews from reviews, in this study, Jieba word segmentation and stop word filtering are applied to these reviews. A hotel review corpus is built, and the BERT model is used to represent the text word vector. Then, a heterogeneous information network *G* = (*V*, *E*) with review text, review topic, and travel types as nodes is constructed as shown in Figure 5, where the node set *V* is *V* = *R*∪*T*∪*P* and the edge set *E* represents the relationship between nodes.

The article "Hotel Review Classification Based on the Text Pretraining Heterogeneous Graph Neural Network Model" was published in 2022. Journal: Comput Intell Neurosci.

For the relationship between reviews and topics, the model adopts the fuzzy matching principle to establish the topic word index of predefined topics, which is shown in Figure 1. If the reviews contain topics, the edge between the topic and the review is constructed. Because each user may mention different aspects of the hotel experience in a review, each review may be linked to multiple topics.

Secondly, the connection between each review and the travel types is established. All users are divided into five categories: solo travel, friends travel, parent-child family travel, couples travel, and business travel. Then, each corresponding review will also be linked to a travel type. Thus, the heterogeneous information network based on hotel review information is established. The purpose is to explore the potential relationship between travel types, user reviews, and review topics through heterogeneous networks, expand text content and semantic features, and provide a basis for mining user preference characteristics and the final classification of reviews.

The heterogeneous information network based on user reviews as shown in Figure 5 enriched the semantic information of hotel reviews and helped improve the classification effect of subsequent reviews. For example, business travelers may pay more attention to the location, transportation, and cleanliness of the hotel, “convenient transportation, clean environment, worthy of recommendation for business travelers.” This review has a rich semantic connection to the topics of location and hygiene, so we can recommend it to business travelers.

For the extraction of user preference features, the model adopts the graph convolution neural network [27] and graph attention mechanism in the solving process, respectively, mining the attention of users of different travel types and the attention of different review texts to the topic words, which is used to express the user preference characteristics. The specific solving process is mentioned in Sections 4.1 and 4.2.

The deep fusion based on pretraining model and heterogeneous graph neural network can complement the advantages of the two models; that is, the vector representation of text is improved and the semantic information of text is expanded. The frame structure of the whole model is shown in Figure 1.

## 4. Model Solution

### 4.1. Heterogeneous Information Network

The heterogeneous information network contains three types of nodes, each of which has a specific feature space, which is described in Figure 2. Based on the inspiration of literature [24, 25], the heterogeneous graph convolution is adopted to complete a different feature mapping.

(1) $$\begin{array}{c} H^{\left(l+1\right)}\sigma \left(\sum_{\tau \in Τ}{\tilde{D}}^{-1/2}A_{\tau }^{\prime }{\tilde{D}}^{-1/2}\cdot H_{\tau }^{\left(l\right)}\cdot W_{\tau }^{\left(l\right)}\right). \end{array}$$

In formula (1), the matrix *A*′ is the node self-connecting adjacency matrix, which is multiplied by its degree matrix ${\tilde{D}}^{-1/2}$ to complete normalization. The rows represent all nodes, and the columns represent adjacent nodes of node type *τ*. Different from graph convolution network (GCN), which is suitable for homogeneous networks, graph convolution neural network is adopted here to map features **H**_*τ*_^(*l*)^ of different types of nodes to the same dimensional space. **W**_*τ*_^(*l*)^ is a trainable transformation matrix considering different node types, and *σ*(·) represents the activation function. In this study, ReLU function is used as the activation function. **H**^(*l*+1)^ is the implicit layer representation of the nodes of layer *l* + 1 in the graph convolutional network. **H**^(0)^ represents the initial features of the node [2].

The article "Hotel Review Classification Based on the Text Pretraining Heterogeneous Graph Neural Network Model" was published in 2022. Journal: Comput Intell Neurosci.

In heterogeneous information networks, two nodes can be connected by different semantic paths, called meta-paths. Under each meta-paths *ϕ*, each node has a set of neighbor node. In order to capture the neighbor nodes structure information and semantic information, as shown in Figure 6, the paper adopted a figure attention mechanism to study the neighbor node weights of the two meta-paths, respectively, and carries on the polymerization to obtain the comment text nodes embedding based the specific semantic.

### 4.2. User Preference Characteristic Extraction Based on the Attention Mechanism

The attention model is widely used in various types of deep learning tasks such as natural language processing, image recognition, and speech recognition, and it is one of the core technologies that deserve the most attention and in-depth understanding in deep learning technology. The essence of the attention mechanism algorithm can also be regarded as the attention distribution coefficient, which calculates the influence of each input item on the output weight.

In the heterogeneous information network based on hotel reviews, each travel type node may be connected with multiple reviews or multiple topics, so it is necessary to distinguish the preference characteristics of each travel type and calculate the attention of each travel type and each review and review topic. The attention mechanism can be introduced to assign different attention values to each node. Given node features as input, the network can learn the attention values between nodes and other nodes through the power mechanism and get the node representation with preference features. This study applies the attention mechanism in three steps:

(1) Define a scoring function:
  (2) $$\begin{array}{c} c_{ij}=a\left(Wt_{i},Wt_{j}\right), \end{array}$$
   where, *t*_*i*_ and **t**_*j*_ represent the feature representation of two different nodes and *a* represents the shared parameter matrix _***W***_ trained by a layer of forward neural network.
(2) It is assumed that node *i* has *k* neighbor nodes. Next, the LeakyReLU activation function is used to map the resulting score to between (−0.2, +*∞*). Finally, the normalized score is performed to obtain the attention coefficient.
  (3) $$\begin{array}{c} \alpha_{\mathrm{ij}}=\frac{\text{exp}\left(\mathrm{Leaky}\left(a^{T}\left[Wt_{i},Wt_{j}\right]\right)\right)}{\sum_{k\in N_{i}}\text{exp}\left(\mathrm{Leaky}\left(a^{T}\left[Wt_{i},Wt_{k}\right]\right)\right)}, \end{array}$$
   where *a*^*T*^ is learnable parameter in the network.
(3) The representation of node *i* of a given meta-path *ϕ* can be obtained by aggregating the projection features of neighbor nodes with corresponding attention vectors.

(4) $$\begin{array}{c} Z_{i}^{\phi }=\sigma \left(\frac{1}{K}\sum_{K=1}^{K}\sum_{j\in N_{i}}\alpha_{ij}W^{k}h_{j}\right). \end{array}$$

Multiple attention mechanism is adopted here, where K is the number of attention mechanism.

The article "Hotel Review Classification Based on the Text Pretraining Heterogeneous Graph Neural Network Model" was published in 2022. Journal: Comput Intell Neurosci.

The node representation under different meta-paths is aggregated and averaged to obtain the final node representation *Z*_*i*_. In the heterogeneous information network built above, the attention mechanism is added to the two different meta-paths respectively, as shown in Figure 6. The attention of the review text itself to the topic words is calculated without considering the travel types, and then, the attention of the reviews of different travel types to the topic words is calculated as shown in Figure 6.

Finally, the user preference characteristics of aggregated travel types and review topics are obtained; that is, the final embedded representation of any review text node is as follows:

(5) $$\begin{array}{c} Z=\sum_{i\in N_{i}}\beta_{i}^{\left(\phi \right)}Z_{i}^{\phi }. \end{array}$$

The final embedding of nodes can complete the node classification task through softmax classifier and identify travel types according to hotel reviews, to provide more suitable review information for users of different travel types. The cross-entropy loss function *L* is used in the model training of multi-objective classification task to optimize the back propagation.

(6) $$\begin{array}{c} L=\frac{1}{N}\sum_{i}\sum_{c=1}^{M}y_{ic}\log\left(p_{ic}\right), \end{array}$$

where *M* is the number of categories. If the true category of sample *i* is equal to *c*, the value of *y*_*ic*_ is equal to 1; otherwise, it is equal to 0. *p*_*ic*_ represents the predicted probability that sample *i* belongs to class *c*.

The article "Hotel Review Classification Based on the Text Pretraining Heterogeneous Graph Neural Network Model" was published in 2022. Journal: Comput Intell Neurosci.

### 4.3. Model Complexity Analysis

The BERT-HGAN model consists of two main parts:

1. BERT pretraining: complexity of BERT model is *O*(*n*^2^ · *d*), *n* is sequence length, and *d* is embedded dimension. Although the model complexity is not very high, large-scale training will increase the model training time. At the same time, the Bert model can obtain results from pretraining of unlabeled datasets, so it can avoid a large number of human annotations and reduce labor costs.
2. Heterogeneous network: the model complexity of heterogeneous network is *O*(|*v*|^2^), where *v* is the number of nodes in the network.

## 5. Experiment and Result Analysis

### 5.1. The Experiment

The classification model selects 50,000 tagged reviews from the corpus as datasets, of which 60% are training sets, 20% are test sets, and 20% are validation sets.

In the model, the parameter values of K are the number of topic words, and we set *K* = 15, which is discussed in Figure 4. We set the layers of the neural network *L* = 2, the dimension of the hidden layer is 512, and the embedded dimension of the pretrained words is 512. In the process of model training, the learning rate was set as 0.005 and the loss rate was set as 0.8.

To verify the effectiveness of the model in this study, the following five models were used as baseline models for comparative experiments.

  BERT: this model is the ablation experiment of the model in this paper, and the word vector obtained by the BERT model is directly added into softmax classifier for classification.
  Heterogeneous graph attention networks (HGANs): this model is also the ablation experiment of the method in this study. Without the Bert word vector training and topic recognition based on fuzzy matching, the heterogeneous network is directly used to classify the text.
  ERNIE2.0 (a continual pretraining framework for language understanding): it is a pretraining framework for semantic understanding based on continuous learning, which uses multitask learning to incrementally construct pretraining tasks.
  TF-IDF + SVM (support vector machine): TF-IDF is used to extract text features, and SVM is used as a classifier for text classification.
  TextCNN (graph convolutional networks for text classification): the model uses the structure of convolutional neural network (CNN) to classify texts.

The article "Hotel Review Classification Based on the Text Pretraining Heterogeneous Graph Neural Network Model" was published in 2022. Journal: Comput Intell Neurosci.

In addition, we validated our model using the other two open datasets.

  THUCNews: generated from historical data of Sina news subscription channels from 2005 to 2011, it contains 740,000 news documents. It includes 14 categories: finance, lottery, real estate, stocks, home, education, technology, society, fashion, politics, sports, horoscope, games, and entertainment.
  Headlines Today News: a total of 382,688 texts are from Headlines Today News, distributed in 15 categories: story, culture, entertainment, sports, finance, house, car, education, technology, military, travel, world, stock, and game.

Similar to the model construction introduced above, in these two news datasets, we built heterogeneous networks with categories, texts, and subject words as nodes and then carried out model training.

Accuracy, recall, and F1 score were selected as three evaluation indexes.

TP means that the prediction result is positive sample (1), which is actually positive sample (1), and the prediction is correct.

FN means that the prediction result is positive sample (1), but actually negative sample (0), so the prediction is wrong.

FP means that the prediction result is negative sample (0), which is actually positive sample (1), and the prediction is wrong.

TN means that the prediction result is negative sample (0), which is actually negative sample (0). The prediction is correct.

(7) $$\begin{array}{c} \mathrm{Precision=}\frac{\mathrm{TP}}{\mathrm{TP+NP}},\\ \mathrm{recall=}\frac{\mathrm{TP}}{\mathrm{TP+FN}},\\ \mathrm{accuracy=}\frac{\mathrm{TP+TN}}{\mathrm{TP+FN+FP+TN}},\\ F_{1}=\frac{2\text{PR}}{P+R}, \end{array}$$

where *R* is the value of recall, and P is the value of precision.

### 5.2. Analysis of User Preferences of Different Travel Types

In the process of solving the above model, GCN is used to complete the feature mapping of different types of nodes. Combined with the attention mechanism, the attention of different review texts to topic words is calculated as shown in Figure 7, and the attention of users of different travel types to different topic words is shown in Figure 8, to mine the potential relationship between review texts and users' travel types and obtain the preference characteristics of users. The color of the theme in the figure indicates the level of attention. The darker the color, the higher the attention.

It can be seen from Figure 8 that different travel types of user reviews pay different attention to the topic of hotel service. Business travelers pay more attention to location, catering, and service. This may be because the users on business trips tend to pay more attention to whether the hotel is closer to the destination and whether the transportation is convenient; in parent-child travel, more attention is paid to whether the room space is large enough, whether children's activities are convenient, and whether there are facilities for children to play, so the topic of room, sanitation, and facilities is relatively high. Friends will pay more attention to the hotel's service, price, and facilities; couples will pay more attention to the decoration of the room, whether there is a smart home; solo travelers pay more attention to hotel prices, hygiene, and room privacy issues.

The article "Hotel Review Classification Based on the Text Pretraining Heterogeneous Graph Neural Network Model" was published in 2022. Journal: Comput Intell Neurosci.

### 5.3. Analysis of Classification Results

It can be seen from Table 2 that the algorithm combining text extraction method and deep learning model proposed in this study has significantly improved the effect compared with SVM + TF-IDF algorithm and TextCNN model. The effect of BERT model alone or HGAN model is far inferior to that of BERT + HGAN model proposed in this study. Compared with BAIDU Wenxin's latest model REIN2.0, the effect is also slightly improved.

In the three datasets, BERT-HGAN model performs better than other models, but compared with the other two datasets, the accuracy of the dataset about hotel reviews is slightly lower, which may be because news texts tend to be described around only one topic, while review texts may involve multiple topics and emotions. This has always been a challenge in the task of classifying review texts.

Figure 9 shows the impact of iteration number on accuracy. It can be found that the accuracy of the model keeps improving with the increase in iteration number. When the iteration number is 400, the model effect reaches the best.

Finally, the influence of the selected number of topic words contained in each category on the accuracy based on the fuzzy matching principle is analyzed as shown in Figure 4.

After setting different values of the topic words related to reviews, the model classification results were compared. When the number of topic words of each topic was 15, the model achieved the best classification effect.

## 6. Conclusion

The user's review information often reflects the real choice and experience of the user. When the user actually conducts the hotel search, the user usually pays special attention to the review written by the user with the same travel demand. Therefore, the review text is closely related to the user's choice preference. The analysis and application of the review text should not only be limited to emotion analysis and hotel management, but also to analyze the review text information, its potential relationship is excavated with user demands and a basis for hotel recommendation is provided.

The article "Hotel Review Classification Based on the Text Pretraining Heterogeneous Graph Neural Network Model" was published in 2022. Journal: Comput Intell Neurosci.

To mine user preference information based on existing reviews, this study first established a super-large hotel review prediction library and combined the advantages of text pretraining and graph neural network algorithms to build a BERT-HGAN model. The BERT model is used to represent the review text with word vector, and the review subject word index is established based on the fuzzy matching rules. Then, a heterogeneous information network with review texts, review topic, and travel types as nodes is established. In addition, a two-force mechanism is added in the network to calculate the attention of topic words in different review texts and the attention of users of different travel types to different topic words. From the perspective that different types of travel users have different demands, the potential relationship between user preference and review text is mined, and travel type preference characteristics are extracted. Finally, a softmax classifier is used for hotel review identification. The results show that the classification accuracy of the proposed model is 70.45%, which is better than the other five comparison models, verifying the effectiveness of the proposed model.

The results of review classification can be presented to users as reasons for hotel recommendation when only the travel types of users are known. Therefore, the model in this study can be applied to the hotel recommendation system to help users make better decisions. Meanwhile, it can also help hotel managers to improve the service quality of hotels.

In future work, the author will continue to consider the influence of other variables such as hotel star, specific location, price, room type, distance, and user attributes on user preference.

## Figures and Tables

**Figure 1:** Structure of the BERT-HGAN model.

**Figure 2:** Flowchart of the BERT-HGAN model.

**Figure 3:** Word cloud of the whole dataset.

**Figure 4:** Influence of the selection of the number of relevant subject words on the results.

**Figure 5:** Heterogeneous graph networks based on user reviews.

**Figure 6:** Attentional mechanisms are applied from two angles.

**Figure 7:** Examples of a review's focus on different subject headings.

**Figure 8:** Users' attention to the topic of different travel types.

**Figure 9:** Effect of iteration number on accuracy.

**Table 1:** Topic words for reviews.

Topic	Topic words
Location	Place, geographical position, geographical environment, geographical location, travel, address, traffic, surrounding environment, close to, downtown, airport, subway, walking, taxi
Catering	Breakfast, food, eat, dinner, lunch, repast, buffet, have a meal, beer and skittles, delicious, cafe, food and beverage, bar, drinks, snacks
Service	Polite, attitude, friendly, enthusiasm, cordial, patience, family, satisfying service, give response to every prayer, personnel quality, hospitality, satisfied, zealous, warmth, smile
Room	Guest rooms, space, room type, toilet, suite, daylight, equipment, smart, area, decorate, curtain, shower, high technology, inside the house, extra bed
Price	Cost, price table, room rate, economical, cost-effective, high-performance cost ratio, cheap, low price, discount, slack season, level, reasonable price, inexpensive, expensive, worthlessness
Cleanliness	Clean, neat, clean and sanitary, salubrious, environment, tidiness, orderliness, exquisite, sweep, brilliancy, smell, peculiar, dirty, sterilize, allergy
Facilities	Billiards, gymnasium, room, swim, running machine, laundry, amusement park, open, installation, instrument, fitness equipment, water quality, swim ring, water sports, billiards, naughty castle.

The article "Hotel Review Classification Based on the Text Pretraining Heterogeneous Graph Neural Network Model" was published in 2022. Journal: Comput Intell Neurosci.

**Table 2:** Comparison of results.

Dataset	Comparative model	Accuracy	Recall	*F*1 score
Hotel review (our dataset)	BERT + HGAN	0.70	0.72	0.72
	BERT	0.62	0.62	0.61
	HGAN	0.51	0.46	0.59
	ERNIE2.0	0.69	0.67	0.68
	TF-IDF + SVM	0.36	0.30	0.33
	TextCNN	0.50	0.50	0.48

THUCNews	BERT + HGAN	0.83	0.84	0.84
	BERT	0.72	0.74	0.68
	HGAN	0.71	0.75	0.73
	ERNIE2.0	0.78	0.74	0.74
	TF-IDF + SVM	0.48	0.66	0.45
	TextCNN	0.57	0.83	0.68

Headlines Today News	BERT + HGAN	0.78	0.76	0.80
	BERT	0.65	0.83	0.62
	HGAN	0.72	0.80	0.68
	ERNIE2.0	0.76	0.88	0.77
	TF-IDF + SVM	0.58	0.67	0.62
	TextCNN	0.65	0.72	0.73

## Data Availability

The data used to support the findings of this study are available from the corresponding author upon request.
